The article "Association between health-enhancing physical activity and the social factors, lifestyle and dietary characteristics" was published in 2024. Journal: PLoS One.

# Association between health-enhancing physical activity and the social factors, lifestyle and dietary characteristics

**DOI:** 10.1371/journal.pone.0311974

**Published:** 2024-11-11

**Authors:** Dragan Djurdjevic, Zorica Terzic-Supic, Jovana Todorovic, Vesna Bjegovic Mikanovic, Aleksandra Radovanovic Spurnic, Ulrich Laaser

**Affiliations:** 1 Department of Sports Medicine, Faculty of Medicine, University of Belgrade, Belgrade, Serbia; 2 Faculty of Medicine, Institute of Social Medicine, University of Belgrade, Belgrade, Serbia; 3 Clinic for Infectious and Tropical Diseases, University Clinical Centre of Serbia, Belgrade, Serbia; 4 Faculty of Medicine, University of Belgrade, Belgrade, Serbia; 5 International Public Health, Faculty of Health Sciences, Bielefeld University, Bielefeld, Germany; Xiamen University - Malaysia Campus: Xiamen University - Malaysia, MALAYSIA

## Abstract

The World Health Organization (WHO) recommends minimum of 150 minutes of moderate intensity aerobic physical activity or 75 minutes of vigorous intensity aerobic physical activity along with at least two sessions of muscle strengthening exercises per week. Compliance with these recommendations is classified as Health Enhancing Physical Activity (HEPA). The aim of this study was to analyze the association between the HEPA and the social factors, lifestyle and dietary characteristics. We conducted the secondary analyses of the data from the Serbian National Health Survey 2019, on 12067 adult participants classified in two groups: with HEPA and without HEPA based on the compliance with the WHO recommendations. Prevalence of HEPA was 3.3% (394/12067). Multivariate logistic regression analysis showed positive association between HEPA and male sex (OR: 4.25, 95% CI: 2.68–6.73), average (OR: 3,01, 95% CI: 1.13–8.04), good (OR: 3.10, 95% CI: 1.21–7.94) and very good (OR: 4.64, 95% CI: 1.82–11.84) income quintile being single (OR: 1.85, 95% CI: 1.16–2.95), the number of portions of fruits per day (OR: 1.29, 95% CI: 1.09–1.53), the frequency fresh fruit/vegetable juice consumption (OR: 1.20, 95% CI: 1.02–1.40), and being non-smoker (OR: 1.67, 95% CI: 1.03–2.73). There was a negative association between HEPA and age (OR: 0.96, 95% CI: 0.95–0.98), BMI (OR: 0.94, 95% CI: 0.88–1.00), average self-rated health (OR: 0.18, 95% CI: 0.12–0.60), and the frequency of non-alcoholic beverages consumption (OR: 0.75, 95% CI: 0.62–0.89). Since only a small percentage of the adult population in Serbia meets the WHO recommendations for physical activity, action is required. This should involve creating future strategies and policies, as well as initiatives focused on education and raising awareness about the importance of physical activity and health.

## Introduction

Physical activity (PA) is one of the most important determinants of health and common part of health promotion activities [1]. It is associated with the improved health and decreased overall mortality [2].

The World Health Organization (WHO) recommends minimum of 150 minutes of moderate intensity aerobic physical activity or 75 minutes of vigorous intensity aerobic physical activity per week along with at least two sessions of muscle strengthening exercises per week [1]. Compliance with these recommendations is classified as Health Enhancing Physical Activity (HEPA) [1]. More than a quarter of adults worldwide, do not meet the recommendation on minimal PA [3], which is associated with the increased prevalence of obesity, cardiovascular diseases, diabetes, cancer, and overall premature mortality [1]. Insufficient PA is associated with the 20–30% increased risk of all-cause mortality, leading to 3.2 million deaths and 32.1 million DALYs (disability-adjusted life years) each year [4].

Studies have shown that there is an association between sex, age, education, income and smoking with the prevalence of sufficient physical activity [5]. Sex differences have been described starting from an early age and tend to persist throughout lifetime, due to different factors including family, environment and entire community [6]. Physical activity has an inverse association with age [6]. Economic factors are associated with the health inequalities, population health and lifestyles in the general population [7, 8]. Income inequalities are especially associated with the increase in prevalence of insufficient physical activity, mainly in high and middle income countries [8].

Being married along with better health status and absence of chronic illnesses have been associated with the sufficient physical activity [5]. Lifestyle characteristics such as smoking status are commonly associated with lower levels of physical activity, while regular breakfast as a part of balanced and diverse diet seems to be associated with higher levels of physical activity [5].

There were numerous public health policies in the past decades aiming to increase the prevalence of HEPA in the European Union countries, as well as to support the compliance with the recommendations among the general population [9–11]. These policies were commonly routed in the sustainability criteria as there is a wide spread belief that there is a overlapping between the sustainable development in general and the health status, specifically healthy lifestyles and physical activity [12]. Majority of the public health policies and programs, even smaller projects, combine the support of individuals’ compliance with the healthy lifestyles and the increase in environmental awareness [13]. The results from the European Health Interview Survey conducted in all European Union countries, and Iceland, Norway, Serbia and Turkey [14] showed the prevalence of HEPA was around 30% [15], however, the factors associated with HEPA are not sufficiently examined so far.

The main hypothesis of this study was that there is an association between the social characteristics, components of the healthy lifestyle (healthy diet, non-smoking, no alcohol consumption) and compliance with HEPA. The aim of this study was to analyze the association between the HEPA and the social factors, lifestyle and dietary characteristics.

## Materials and methods

This was a secondary analysis of the data from the Serbian National Health Survey from 2019, which included total of 15621 participants. Our analysis included total of 12067 participants, older than 18 years of age. The study was conducted between the October and December 2019.

The target population of the Serbian National Health Survey included the residents of Serbia, older than 15 years, who were not living in any form of the institutional housing. The participants living in collective housing (students’ dorms, institutions for children with developmental problems, elderly homes, monasteries, etc.) were, therefore, excluded from the study.

The sample was two-step cluster sample. The random sample from census circles (cluster of households) was chosen, in proportion to its size, and then in the second step, the sample of households was chosen randomly from each cluster. The sample size was calculated based on the study power and in order to allow for assessment of the standard error. The sample size was set at 6000 households. The total of 10 households was randomly chosen from each of the census circles, meaning that the study included the total of 600 census circles. The number of participants in each region was determined proportionally based on the number of residents in the last census. All the residents in the selected households (older than 5 years) were included in the Serbian National Health Survey. The participants were given both oral and written explanation about the study, its processes and aims and all participants provided written consent to participate in the study. This analysis was approved by the Ethical Committee of the Faculty of Medicine, University of Belgrade (No. 1322/VII-3 from 07.07.2022).

The instrument used for the Serbian National Health Survey is the European Health Interview Survey (EHIS). The data was gathered using the face-to-face interview, self-reported questionnaires and measurements of the anthropometric characteristics of the participants (height, weight, and arterial blood pressure).

The data gathered referred to the participants’ sex (female or male), age (in years), body mass index (calculated based on the measurement of height and weight as BMI = weight in kilograms/ (height in meters)^2^), marital status (married/in a relationship or single), income quintiles (self- reported as very poor, poor, average, good, very good), educational level (reported as the highest educational level achieved: primary, secondary, tertiary), employment status (defined as employed or inactive- student, retired, housewife, unemployed), self-rated health (as poor, average, good), presence of chronic illness (yes/no), social support (measured as the number of people that the participant can turn for help to).

The lifestyle characteristics examined were the physical activity, dietary characteristics, smoking, and alcohol use. Physical activity was examined using the EHIS-PAQ questionnaire, the short, specific questionnaire, which was used in the population surveys before [16] and is considered to be easily understandable while being easy to complete. The EHIS-PAQ allows the examination of the work-related PA, transportation-related PA, leisure PA, health- enhancing PA (HEPA) and muscle-strengthening PA [17]. HEPA calculation is based on the recommendation from the World Health Organization that states that the adults, aged 18 years or older should have aerobic PA within 150–300 minutes of moderate intensity, or 75–150 minutes of vigorous aerobic PA, or the combination of moderate and vigorous intensity per week, along with at least two sessions of muscle-strengthening PA per week [1]. For the calculation of the HEPA we used the information on the transport-related PA and on the leisure-time PA combined. As it was shown in the previous studies, self-reported moderate PA is strongly associated to the objective measurements when walking is excluded. Thus, we excluded walking from the calculations for the moderate intensity aerobic PA [16].

The dietary characteristics of the participants were examined using the EHIS dietary questionnaire [18]. For this study we analysed number of portions of fruits per day, number of portions of vegetables per day, the frequency of consumption of fresh fruit/vegetable juice and the frequency of consumption of non-alcoholic beverages [19]. Alcohol consumption was defined as reported consumption of any alcoholic drinks in the past year. Smoking was examined as current smoking (yes/no). Heavy episodic drinking was defined as a consumption of six or more alcoholic beverages in one occasion.

Based on the calculated HEPA participants were classified in two groups: participants with HEPA (117) and participants without HEPA (11913). Total of 21 variables were analyzed, and these were: sex, age, BMI, marital status, income quintiles, educational level, employment, general health, chronic illness, social support, aerobic PA, work-related PA, the number of portions of fruits daily, the number of portions of vegetables or salads daily, the frequency of fresh fruit/vegetable juice consumption, the frequency of non-alcoholic beverages consumption, smoking, alcohol consumption, and heavy episodic drinking in the past year (6 or more drinks).

The statistical analyses were done using the descriptive and analytical statistics. The differences between the categorical variables were examined using the Chi-square test. The differences between the groups on the numerical variables were assessed using the T-test for the variables with the normal distribution and with Kruskal Wallis test for the variables without the normal distribution. The normality was examined using the Kolmogorov-Smirnov test. All the variables which were shown to be significant were entered in the multivariate logistic regression analysis (MLRA) with HEPA as an outcome variable. We presented Odds Ratios (ORs) and 95% Confidence Intervals (95% CIs). Model fit was assessed using Nagelkerke R square. The effect size was calculated using the Cramer’s V for Chi-square test (small-0.07, medium-0.21, large-0.35) and Cohen’s D for T-test (small-0.20; medium-0.50; large- 0.80). The statistical significance was considered as p<0.05. All statistical analyses were done using the Statistical Software for Social Sciences SPSS 22.0.

## Results

The response rate was 84.4% (13178/15621). Total of 394 (3.3%) participants reported HEPA. The participants with HEPA were more frequently male (75.6% vs. 24.4%), with lower average age (35.99±15.33 vs. 53.96±17.42 years), BMI (24.55±3.09 kg/m^2^ vs. 26.15±4.52 kg/m^2^), and more frequently single (66.2% vs. 36.4%), had significantly higher frequency of very good income (32.5% vs. 18.5%), good general health (94.7% vs. 61.8%), tertiary education (37.6% vs. 18.05), lower frequency of chronic illnesses (16.3% vs. 48.5%), and higher social support. The socio-demographic, socio-economic and health status characteristics of the participants are presented in Table 1.

**Table 1:** Socio-demographic, socio-economic characteristics and health status of the participants with and HEPA.

Characteristics	Total	With	Without	p-value	ES
	N (%)	HEPA	HEPA		
		N (%)	N (%)		
Sex					
Male	5834 (48.3)	298 (75.6)	5536 (47.4)	**<0.001**	0.10 (small)
Female	6233 (51.7)	96 (24.4)	6137 (52.6)		
Age in years (X±SD)	53.19±17.71	35.99±15.33	53.96±17.42	**<0.001**	1.06 (large)
BMI in kg/m^2^ X±SD	26.08±4.48	24.55±3.09	26.15±4.52	**<0.001**	0.38 (small)
Marital status					
Married/ in a relationship	7544 (62.6)	133 (33.8)	7411 (63.6)	**<0.001**	0.11 (small)
Single	4501 (37.4)	261 (66.2)	4240 (36.4)		
Income quintiles					
Very poor	2432 (20.2)	45 (11.4)	2387 (20.4)	**<0.001**	0.07 (small)
Poor	2437 (20.2)	51 (12.9)	2386 (20.4)		
Average	2472 (20.5)	80 (20.3)	2392 (20.5)		
Good	2434 (20.2)	90 (22.8)	2344 (20.1)		
Very good	2292 (19.0)	128 (32.5)	2164 (18.5)		
Educational level					
Primary	2955 (24.5)	26 (6.6)	2929 (25.1)	**<0.001**	0.10 (small)
Secondary	6861 (56.9)	220 (55.8)	6641 (56.9)		
Tertiary	2247 (18.6)	148 (37.6)	2099 (18.0)		
Employment					
Employed	7595 (63.0)	201 (51.1)	7394 (63.4)	**<0.001**	0.04 (small)
Inactive (unemployed, student, retired, housewife)	4453 (37.0)	192 (48.9)	4261 (36.6)		
General health					
Poor	1452 (12.0)	5 (1.3)	1447 (12.4)	**<0.001**	0.12
Average	3032 (25.1)	16 (4.1)	3016 (25.8)		
Good	7580 (62.8)	372 (94.7)	7208 (61.8)		
Chronic illness					
Yes	5718 (47.4)	64 (16.3)	5654 (48.5)	**<0.001**	0.11 (small)
No	6338 (52.6)	329 (83.7)	6009 (51.5)		
Social support					
No one	254 (2.1)	3 (0.8)	251 (2.2)	**<0.001**	0.07 (small)
1–2 people	3995 (33.2)	72 (18.3)	3923 (33.7)		
3–5 people	5602 (46.6)	203 (51.5)	5399 (46.4)		
6 or more people	2176 (18.1)	116 (29.4)	2060 (17.7)		

HEPA, health-enhancing physical activity; BMI, body mass index; ES, effect size.

*effect size was calculated using Cramer’s V (df-2) for Chi-square; Cohen’s d for T-test.

The participants with HEPA had higher average number of portions of fruit per day (2.12±1.51 vs. 1.73±0.94), higher average number of portions of vegetables or salad per day (2.17±1.21 vs. 1.93±1.01), higher frequency of fresh fruit/vegetable juice consumption daily, higher frequency of daily consumption of non-alcoholic beverages, higher frequency of alcohol consumption (67.4% vs. 47.0%), lower frequency of participants who never engaged in binge drinking (41.8% vs. 51.1%), and lower frequency of smoking (23.1% vs. 32.1%). Differences in the lifestyle and dietary habits of the participants are presented in Table 2.

**Table 2:** Lifestyle and dietary habits among the participants with and without HEPA.

Characteristics	Total	With	Without	p-value	ES
	N (%)	HEPA	HEPA		
		N (%)	N (%)		
Aerobic PA in minutes per week (X±SD)	83.68±195.73	475.43±402.22	66.06±159.94	**<0.001**	2.41 (large)
Work-related PA					
Light physical effort	4715 (39.1)	156 (39.6)	4559 (39.1)	0.057	0.06 (small)
Moderate physical effort	5745 (47.7)	198 (50.3)	5547 (47.6)		
Heavy physical effort	1239 (10.3)	37 (9.4)	1202 (10.3)		
No	355 (2.9)	3 (0.8)	352 (3.0)		
Number of portions of fruits, excluding juices per day X±SD	1.75±0.97	2.12±1.51	1.73±0.94	**<0.001**	0.34 (small)
Number of portions of vegetables or salad, excluding juices and potatoes per day X±SD	1.94±1.02	2.17±1.21	1.93±1.01	**<0.001**	0.21 (small)
Frequency of fresh fruit/vegetable juice consumption per day					
Never	3527 (29.3)	72 (18.3)	3455 (29.7)	**0.001**	0.07 (small)
Less than once a week	4124 (34.2)	107 (27.2)	4017 (34.5)		
1–3 times per week	2748 (22.8)	124 (31.5)	2654 (22.5)		
4–6 times per week	1022 (8.5)	56 (14.2)	966 (8.3)		
Once per day or more	620 (5.1)	35 (8.9)	585 (5.0)		
Frequency of non-alcoholic beverages consumption per day					
Never	2931 (24.3)	105 (26.6)	2826 (24.2)	**0.045**	0.03 (small)
Less than once a week	3522 (29.2)	108 (27.4)	3414 (29.3)		
1–3 times per week	3081 (25.6)	83 (21.1)	2998 (25.7)		
4–6 times per week	1497 (12.4)	52 (13.2)	1445 (12.4)		
Once per day or more	1020 (8.5)	46 (11.7)	974 (8.4)		
Smoking					
Yes	2784 (31.8)	67 (23.1)	2717 (32.1)	**0.001**	0.03 (small)
No	5966 (68.2)	223 (76.9)	5743 (67.9)		
Alcohol consumption					
Yes	3923 (47.7)	194 (67.4)	3729 (47.0)	**<0.001**	0.07 (small)
No	4293 (52.3)	94 (32.6)	4199 (53.0)		
Heavy episodic drinking every month in the last year (6 or more drinks)					
Yes in a year, but not in a month	1004 (27.6)	62 (33.7)	942 (27.3)	**0.045**	0.04 (small)
Yes, in a month	789 (21.7)	45 (24.5)	744 (21.6)		
No	1839 (50.6)	77 (41.8)	1762 (51.1)		

HEPA, health-enhancing physical activity; PA, physical activity; ES, effect size.

*effect size was calculated using Cramer’s V (df-2) for Chi-square; Cohen’s d for T-test.

Multivariate logistic regression analysis showed that health-enhancing PA was associated with male sex (OR: 4.25, 95% CI: 2.68–6.73), age (OR: 0.96, 95% CI: 0.95–0.98), average, good and very good self rated financial status (OR: 3.01, 95% CI: 1.13–8.04; OR: 3.10, 95% CI: 1.21–7.94; OR: 4.64, 95% CI: 1.82–11.84), average self-rated health (OR: 0.18, 95% CI: 0.52–0.60), being single (OR: 1.85, 95% CI: 1.16–2.95), the number of portions of fruits per day (OR: 1.29, 95% CI: 1.09–1.53), the frequency fresh fruit/vegetable juice consumption (OR: 1.20, 95% CI: 1.02–1.40), the frequency of non-alcoholic beverages consumption (OR: 0.75, 95% CI: 0.62–0.89), and being non-smoker (OR: 1.67, 95% CI: 1.03–2.73). Nagelkerke R square for the model fit summary was 0.268. The results of the multivariate logistic regression analysis with HEPA as an outcome variable are shown in Table 3.

**Table 3:** Multivariate logistic regression analysis with HEPA as an outcome variable.

Characteristics	OR (95% CI)	ES
Sex		
Male	**4.25 (2.68–6.73)**	Medium
Female	1.0 reference category	
Age	**0.96 (0.95–0.98)**	Small
BMI	**0.94 (0.88–1.00)**	Small
Income quintiles		
Very poor	1.0 reference category	
Poor	2.26 (0.82–6.22)	/
Average	**3.01 (1.13–8.04)**	Medium
Good	**3.10 (1.21–7.94)**	Medium
Very good	**4.64 (1.82–11.84)**	Large
Educational level		
Primary	1.0 reference category	
Secondary	1.59 (0.65–3.92)	/
Tertiary	1.91 (0.74–4.92)	/
Employment		
Employed	0.70 (0.45–1.06)	/
Inactive (unemployed, student, retired, housewife)	1.0 reference category	
General health		
Poor	0.58 (0.16–2.09)	/
Average	**0.18 (0.52–0.60)**	Large
Good	1.0 reference category	
Marital status		
Married/ in a relationship	1.0 reference category	
Single	**1.85 (1.16–2.95)**	Small
Social support		
No one	1.0 reference category	
1–2 people	1.18 (0.14–9.63)	/
3–5 people	0.66 (0.35–1.23)	/
6 or more people	0.83 (0.54–1.27)	/
Number of portions of fruits per day	**1.29 (1.09–1.53)**	Small
Number of portions of vegetables per day	1.10 (0.90–1.34)	/
Frequency of fresh fruit/vegetable juice consumption	**1.20 (1.02–1.40)**	Small
Frequency of non-alcoholic beverages consumption	**0.75 (0.62–0.89)**	Small
Smoking		
Yes	1.0 reference category	
No	**1.67 (1.03–2.73)**	Small
Alcohol consumption		
Yes	1.0 reference category	
No	0.85 (0.56–1.29)	/

HEPA, health-enhancing physical activity; BMI, body mass index; ES, effect size.

## Discussion

The aim of this study was to examine the association between the HEPA and the social factors, lifestyle and dietary characteristics. The results of this study showed that the prevalence of HEPA in adults in Serbia was only 3.3%, the third lowest in Europe after Turkey and Romania. The average prevalence of HEPA in Europe in 2019 was 13.6%, ranging from 1.2% in Turkey to 40.1% in Iceland [20]. However, Serbia has not developed the policy aiming to improve physical activity in the general population, unlike many European countries [10], and the development of these policies can influence the physical activity practices in our country. Multivariate logistic regression analysis showed the positive association of HEPA with male sex, income, being single, number of portions of fruits per day, the frequency of fresh fruit/vegetable juice consumption, and being non-smoker. Multivariate logistic regression analysis showed the negative association of HEPA with age, BMI, average general health compared to good health, and the frequency of non-alcoholic beverages consumption. The goodness of fit of the model was examined using the Nagelkerke R square, which was 0.268. As this was the population based study, and the examined factors could not be controlled as it would be in an experimental environment, the R square value was acceptable [21].

Our research indicates that men are about 4 times more likely to engage in HEPA compared to women, a trend also noted across multiple studies, highlighting a significant disparity between males and females in various age groups and settings [22–24]. Among European countries, the largest disparities were observed in Spain, Slovenia, and Ireland, ranging from 10% to 11.4%, while the smallest gaps, between 2.2% and 3.9%, were in Denmark, Turkey, Finland, Iceland, and Poland [12]. Women are less physically active than men throughout the lifespan, starting from early development through infanthood, childhood, adolescence to adulthood [25–28]. These difference may be important from the public health perspective as insufficient physical activity is associated with the increased risks for chronic non-communicable diseases, that are especially prevalent in the past decades [29, 30]. The improvement of physical activities among women and girls can improve their self-confidence and self-esteem, redefine gender roles and provide numerous social and psychological benefits along with the benefits for physical health. It is thought that higher inclusion of women and girls in physical activities can further promote sexual and reproductive health, the increase in self-esteem could decrease sexual harassment and higher self-confidence can lead to more women engaging in leadership, all together leading to more gender equality [31].

We found the association between HEPA and age, as HEPA tends to decrease with the increasing age, as was shown in other European countries, except in Denmark where the level of HEPA does not decrease with age [32]. Our study also showed the association between BMI and HEPA, as with each increase in BMI of 1 kg/m^2^, there was a 6% lower likelihood to be in HEPA group, which was in accordance with previous studies [33]. Participants with average, good and very good self-reported financial status were about 3–4.5 times more likely to have HEPA as showed in some other studies [34–37], although this association is not always linear, as often, higher socio-economic status is associated with more time spent in work-related sedentary activities [37]. People with lower income often do not have enough leisure time and therefore may struggle to meet physical activity recommendations even if they have physically demanding job [38]. On the other hand, among those with high socioeconomic status, physical activity is promoted due to sedentary work behavior [39]. Lower socioeconomic status is often associated with lack of green spaces in the neighborhoods and insufficient opportunities for physical activity [12]. Contrary, higher socioeconomic status is associated with the higher levels of life-satisfaction and higher levels of pro-environmental behaviors [40, 41].

Our study showed that participants with average general health were more than five times less likely to have HEPA than adults with good general health. This was expected as meeting the recommendations for physical activity may be associated with better self-perceived health status [42]. Our study revealed that single participants were 1.85 times more likely to engage in HEPA compared to those who are married or in a relationship, consistent with findings from a study in Poland, Brazil and Pakistan [43–45]. Single individuals might have more flexible schedules, providing more opportunities for physical activities, fewer family-related responsibilities and social motivations to engage in physical activities [43]. Some other studies, reported higher levels of active transportation among single people than those in relationships, as these activities typically require more time than driving, giving single adults an advantage [46, 47]. Furthermore, single people might seek social connections and support through physical activities.

Each additional portion of fruits consumed per day, was associated with 29% increase in the likelihood of having HEPA in our study. Consuming fruits regularly fits into healthy diet [48]. Healthy diet and PA have been linked to health benefits in adults [49] and it was previously shown that health promoting behaviors tend to cluster and are commonly occurring together [50]. Increase in frequency of the fresh fruit/vegetable juice consumption was associated with 1.2 times higher likelihood for HEPA in our study. Drinking fresh fruit juice is considered a part of balanced and diverse dietary habits and is commonly associated with the higher intake of essential nutrients and can reduce risk of being overweight or obese by 22% and of having metabolic syndrome by 27% [51]. We have examined the fruit and vegetable consumption in association with the HEPA as diet with low content of fruit and vegetables is recognized risk factor for numerous chronic illnesses that are the main contributors to population morbidity and mortality such as cancers and cardiovascular diseases, as fruit and vegetables are rich in essential micronutrients, like minerals, vitamins and phytochemicals [52].

Our results showed the increase in frequency of consumption of non- alcoholic beverages was associated with the 25% decrease in likelihood for HEPA. In contrast, study by Werneck et al. showed that non-alcoholic beverages consumption was not associated with PA [53]. In this study we do not have data on daily water intake, so an increase in the frequency of consumption of non-alcoholic beverages may be due to insufficient water intake, which was in the study by Ortuño-Soriano et al showed to be associated with lower PA [54].

Non-smoking status was associated with 1.67 times higher likelihood of HEPA in our study, as well as in the study by Salin et al. who showed that those who are physically active smoke less than those who are not sufficiently active, and that an active lifestyle could prevent smoking [55]. The study by Newsom et al. showed that there is no association between smoking status and PA [56]. Smoking has been a significant public health issue in Serbia for decades, with high prevalence in adults [18, 57, 58] and can be seen as a factor that has influenced the high prevalence of non-communicable diseases in Serbia [59].

To the best of our knowledge, this is the first study examining the association between HEPA and social and lifestyle characteristics in a Balkan country. Moreover, we analyzed the data from the EHIS that was conducted on a representative sample of adults residing in Serbia and with the same methodology as in other European countries, allowing for the comparability of the results. Having in mind such a high prevalence of smoking in a general population in Serbia (as well as in other Balkan countries) and the negative association of smoking with physical activity, public health professionals seem to have double fold challenge in preserving the population health and in decreasing the prevalence of non-communicable diseases associated with both smoking and insufficient physical activity. This can guide policymakers, not only in Serbia, but throughout the region.

This study has a few possible limitations. This was the cross-sectional study, and we were not able to determine the direction of the association between factors. It is possible that HEPA led to greater awareness of a healthier lifestyle. Further, self-reported questionnaires were used in this research, and results should be interpreted with caution, since participants could report overestimated or underestimated data of their levels of PA and dietary intake.

## Conclusions

Our study identified several significant independent factors associated with HEPA in Serbian adults. Those factors are: male sex, age, BMI, income, general health, being single, number of portions of fruits per day, the frequency of fresh fruit/vegetable juice consumption, the frequency of non-alcoholic beverages consumption, and being non-smoker. Based on the obtained results and an extremely small percentage of the adult population in Serbia who meet the WHO recommendations, an urgent action making future strategies and policies is needed, along actions aimed at education and raising awareness about physical culture and health in general.
